# Xin-Ji-Er-Kang Alleviates Isoproterenol-Induced Myocardial Hypertrophy in Mice through the Nrf2/HO-1 Signaling Pathway

**DOI:** 10.1155/2022/7229080

**Published:** 2022-08-22

**Authors:** Ting-Ting Yu, Li-Jun Sun, Chen Chen, Zi-Jian Wang, Xue-Sheng Liu, Feng-Qin Zhu, Shan Gao

**Affiliations:** ^1^Department of Functional Experiment Training Center, Basic Medical College, Wannan Medical College, Wuhu 241002, China; ^2^Department of Pharmacology, Basic Medical College, Anhui Medical University, Hefei 230032, China; ^3^Anhui Medical University Clinic Medical School of Medicine, Hefei 230032, China; ^4^Department of Anesthesiology, The First Affiliated Hospital of Anhui Medical University, Hefei 230032, China; ^5^Cancer Hospital, Chinese Academy of Science, Hefei 230032, China

## Abstract

Xin-Ji-Er-Kang (XJEK) inhibited cardiovascular remodeling in hypertensive mice in our previous studies. We hypothesized that XJEK may prevent isoproterenol (ISO)-induced myocardial hypertrophy (MH) in mice by ameliorating oxidative stress (OS) through a mechanism that may be related to the nuclear factor erythroid 2-related factor 2 (Nrf2)/heme oxygenase-1(HO-1) pathways. Forty SPF male Kunming mice were randomized into 5 groups (*n* = 8 mice per group): control group, MH group, MH + different doses of XJEK (7.5 g/kg/day and 10 g/kg/day), and MH + metoprolol (60 mg/kg/day). On the eighth day after drug treatment, electrocardiogram (ECG) and echocardiography were performed, the mice were sacrificed, and blood and heart tissues were collected for further analysis. XJEK administration markedly ameliorated cardiovascular remodeling (CR), as manifested by a decreased HW/BW ratio and CSA and less collagen deposition after MH. XJEK administration also improved MH, as evidenced by decreased atrial natriuretic peptide (ANP), brain natriuretic peptide (BNP), and *β*-myosin heavy chain (*β*-MHC) levels. XJEK also suppressed the decreased superoxide dismutase (SOD) and catalase (CAT) activities and increased malondialdehyde (MDA) levels in serum of mice with MH. XJEK-induced oxidative stress may be related to potentiating Nrf2 nuclear translocation and HO-1 expression compared with the MH groups. XJEK ameliorates MH by activating the Nrf2/HO-1 signaling pathway, suggesting that XJEK is a potential treatment for MH.

## 1. Introduction

Myocardial hypertrophy is characterized by myocyte hypertrophy, fibroblast activation, and extracellular matrix accumulation, an adaptive response to processes such as mechanical and neurohumoral stimulation [1]. It is strongly associated with an increased risk of many cardiovascular diseases, such as heart failure, sudden death, and arrhythmia [2]. Sympathetic nerve activation is considered one of the main causes of myocardial hypertrophy. Activation of the *β*-adrenergic receptor is an important contributor to sympathetic nerve excitation, and it is closely related to heart function. Isoproterenol (ISO), a nonselective *β*-adrenergic receptor agonist, has been reported to induce cardiac hypertrophy and is recognized as one of the classic animal models [3]. Recently, many studies have found that sympathetic stress is often associated with increased levels of reactive oxygen species (ROS). Oxidative stress has been identified as one of the key factors contributing to the development of cardiac hypertrophy [4].

The Nfe2l2 gene encodes nuclear factor erythroid 2-related factor 2 (Nrf2), a transcription factor responsible for regulating the cellular redox balance and protective antioxidant and phase II detoxification responses in mammals [5]. In the physiological state, Nrf2 is bound to Kelch-like ECH-associated protein 1 (Keap1), which functions as a negative regulatory factor of Nrf2 and localizes in the cytoplasm, where it activates the process of ubiquitin-mediated degradation. Following oxidative or electrophilic stress, the Keap1 protein dissociates from Nrf2, leading to Nrf2 translocation into the nucleus and the production of antioxidant enzymes such as catalase, glutathione (GSH), superoxide dismutase (SOD), and heme oxygenase-1 (HO-1) [6–8]. As a member of the heme oxygenase family, HO-1 plays a vital role in anti-inflammatory, antioxidant, and antiapoptotic processes [9]. The Nrf2/HO-1 signaling pathway has been recognized as important for the oxidative stress response [10]. Likewise, the Nrf2/HO-1 signaling pathway was reported to exert a protective effect on cardiovascular diseases, such as atherosclerosis, hypertension, heart failure, and ischemia/reperfusion injury [11–14]. However, researchers have not clearly determined whether the changes in the expression levels of Nrf2/HO-1 occur in myocardial hypertrophy induced by ISO.

Xin-Ji-Er-Kang (XJEK) is a Chinese herbal formula that consists of fourteen types of herbs, such as *Panax ginseng* C. A. Mey, *Astragalus mongholicus* Bunge, *Polygonatum odoratum* (Mill.) Druce, *Ophiopogon japonicus* (Thunb.) Ker-Gawl, and so on (Table 1). Clinical and experimental data indicate that XJEK is an effective treatment for hypertension, viral myocarditis, myocardial infarction, and cardiovascular remodeling [15–18]. We have previously shown the protective effect of XJEK on ISO-induced ventricular remodeling in mice, which may be related to its actions in reducing oxidative stress and improving the antioxidant activity in the body [19]. The aims of this research, therefore, are to reveal whether XJEK prevents ISO-induced myocardial hypertrophy and the potential molecular mechanisms, with a focus on the Nrf2/HO-1 signaling pathway.

## 2. Materials and Methods

### 2.1. Animals and Chemicals

Forty male Kunming mice (SPF, 26 ± 2 g) were obtained from Shanghai Slac Laboratory Animal Corp., Ltd. (certificate number: SCXK (JING) 2019–0010) and housed under specific pathogen-free (SPF) conditions (24 ± 2°C, a relative humidity of 60 ± 10%, and alternating 12 h dark/night cycles). All procedures were performed in accordance with the protocol outlined in the Guide for the Care and Use of Laboratory Animals published by the US National Institute of Health (NIH publication no. 85–23, revised 1996) and approved by the Committee on the Ethics of Animal Experiments of Anhui Medical University. XJEK was acquired from the Hefei Seven Star Medical Science and Technology Company (Hefei, China), ISO was purchased from Shanghai Hefeng Pharmaceutical Co., Ltd. (Shanghai, China, 41200801), and metoprolol was obtained from AstraZeneca Pharmaceutical Co., Ltd. (Wuxi, China, 2103070).

### 2.2. Laboratory Animal Grouping and Handling

After one week of adaptive feeding, the animals were randomly divided into the five groups (*n* = 8 mice per group): the control group was fed a standard diet alone; the model group received ISO (2 mg/kg/day) by subcutaneous injection twice a day for 7 days; mice in the XJEK low-dose group were intragastrically administered XJEK (7.5 g/kg/day) beginning on the first day after the subcutaneous injection of ISO; mice in the XJEK high dose group were intragastrically administered XJEK (10 g/kg/day) beginning on the first day after the subcutaneous injection of ISO; and mice in the metoprolol group were intragastrically administered metoprolol (60 mg/kg/day) beginning on the first day after the subcutaneous injection of ISO. All mice were sacrificed after electrocardiogram (ECG) and echocardiography were conducted on the 8th day, followed by the collection of serum and hearts for further analysis.

### 2.3. Measurement of ECG

The BL-420S biological functional experimental system was used to monitor and record the ECGs with standard limb lead II, as described previously [20]. The height and width of the P, T, S waves, QT interval, and P-R interval at baseline and on the 8th day were measured using image analysis software.

### 2.4. Echocardiography

Transthoracic echocardiography was performed using VINNO 6vet (Feiyinuo Technology Co., Ltd., Suzhou, China) following ECG detection. Echocardiographic parameters, including the ejection fraction (EF), fractional shortening of left ventricular diameter (FS), left ventricular posterior wall thickness at end-diastole (LVPWd), left ventricular posterior wall thickness at end-systole (LVPWs), left ventricular diameter at end-diastole (LVIDd), left ventricular diameter at end-systole (LVIDs), left ventricular volume at end-diastole (LVEDv), and left ventricular volume at end-systole (LVESv), were determined.

### 2.5. Collection of Serum and Cardiac Tissues

After color Doppler ultrasound of the heart, 1-2 ml blood samples were collected from the abdominal aorta and centrifuged at 3500 r/min for 10 minutes at 4°C; then, the serum was stored at −80°C until further analysis. Hearts and lungs were collected and irrigated with an ice-cold physiological saline solution. Organ indices were calculated, such as the heart weight/body weight (HW/BW) and lung weight/body weight (LW/BW). The hearts of some mice were incubated with 10% neutral buffer formalin for pathological detection, and the hearts from the remaining mice were stored in a −80°C freezer until further analysis.

### 2.6. Histological Analysis

After 24 hours of fixation, the apex of the mouse heart was dehydrated and embedded in paraffin. Hematoxylin-eosin (HE) and Masson's trichrome staining were applied to observe the prepared 5 *µ*m paraffin sections. Then, images were captured and analyzed with a glass scanner (Pannoramic MIDI, 348, Hungary). The quantitative analysis was conducted by three independent observers using ImageJ software.

### 2.7. Measurement of Serum Superoxide Dismutase (SOD), Malondialdehyde (MDA), and Catalase (CAT) Levels

The serum levels of SOD, MDA, and CAT were measured (reported as U/ml or nmol/ml of serum) using the xanthine oxidase method, thiobarbituric acid reactive substances assay, and ammonium molybdate method, respectively (Jiancheng Institute of Bioengineering Company, Nanjing, China). All measurements were performed according to the manufacturers' protocols.

### 2.8. Western Blot Analysis

A nuclear extraction kit (BestBio, Shanghai, China) was used to extract nuclear proteins from the heart according to the manufacturer's protocol. The protein concentration was measured using a bicinchoninic acid assay (BCA) kit (Jiancheng Institute of Bioengineering Company, Nanjing, China). Total and nuclear proteins derived from the heart tissues were separated on 10%–12% SDS-PAGE gels and transferred to PVDF membranes using the wet transfer method. After blocking with a 5% nonfat milk solution at 4°C for 2 h on a shaker, the membranes were incubated with the following primary antibodies in TBS-T overnight at 4°C: rabbit anti-rabbit Nrf2 (dilution 1 : 800, Abcam, USA) and HO-1 (dilution 1 : 25000, Abcam, USA). After incubation with secondary antibodies (goat anti-rabbit IgG, 1 : 10000; Boster, China), protein expression was detected using a super signal enhanced chemiluminescence (ECL; Amersham Biosciences, Little Chalfont, UK) detection system. The band intensities were analyzed using ImageJ software. GAPDH (dilution 1 : 25000, Affinity, USA) and histone H3 (dilution 1 : 1500, Affinity, USA) protein served as loading controls for the target proteins.

### 2.9. Real-Time Quantitative PCR

Total RNA was extracted from the mouse myocardial tissues using TRIzol reagent. The RNA concentration and purity were determined by measuring the ratio of absorbance at 260/280 using a DS-11 spectrophotometer (Denovix, USA). Total RNA (0.5 *µ*g) was used for RT with the RevertAid First Strand cDNA Synthesis Kit (lot. 01076664; Thermo Scientific), according to the manufacturer's protocol. RT-qPCR SYBR Premix Ex Taq kit (TaKaRa, Dalian, China) was used to determine the expression levels of mRNAs with a Bio-Rad CFX96 real-time PCR detection system. Relative gene expression was normalized to GAPDH. The nucleotide sequences of the primers used are given in Table 2.

### 2.10. Data and Statistical Analysis

The results are presented as the means ± standard deviations (SD). Student's *t*-test was employed for comparisons between two groups. Statistical analyses were performed using SPSS 22.0 software. Results with a *p* value less than 0.05 were considered significant.

## 3. Results

### 3.1. XJEK Ameliorated Cardiac Remodeling in Mice with MH

Morphological hypertrophy of the heart was determined by measuring an increase in the HW/BW ratio. The HW/BW ratio in the model group was significantly increased compared with that in the control group (Figure 1(a)-1(b), *p* < 0.01). In addition, MH caused a significant increase in LW/BW, whereas XJEK (10 g/kg/d) treatment markedly decreased the LW/BW (Figure 1(c), *p* < 0.05).

Based on the histological assessments, the myocardial fibers and myocardial cells in the XJEK and metoprolol-treated groups were arranged in a normal pattern with clear structures and were similar to those in the control diet group. In addition, the myocardial cells in mice from the ISO subcutaneous injection group were loosely and irregularly arranged, exhibiting hypertrophy, and tissue fibrosis was aggravated. These changes were significantly ameliorated by the XJEK treatment and the positive control drug metoprolol (Figure 2, *p* < 0.05).

### 3.2. XJEK Improved Electrocardiography Parameters

The ECG analysis showed a prolonged QT interval, increased R amplitude, and increased heart rate (Figure 3, *p* < 0.01) in the ISO-induced MH group. All these ECG changes in the hypertrophic heart indicate the presence of cardiac ventricular hypertrophy and tachycardia. XJEK and metoprolol administration normalized these electrocardiac abnormalities in mice.

### 3.3. XJEK Improved Heart Function in Mice with ISO-Induced MH

Echocardiography is considered a first-line imaging method for evaluating cardiac function both in the clinic and in mouse models. As shown in Figures 4(a) –4(g), significant increases in EF and FS and decreases in LVESV, LVIDS, LVPWd, and LVPWs were observed in mice treated with XJEK and metoprolol compared to those in mice with MH, suggesting that XJEK and metoprolol injections prevented the development of ISO-induced cardiac hypertrophy and preserved cardiac function.

### 3.4. XJEK Reduced Oxidative Stress in Mice with ISO-Induced MH

A significant increase in serum MDA levels (Figure 5(a), *p* < 0.01) and a decrease in the levels of endogenous cardiac antioxidants such as SOD (Figure 5(b), *p* < 0.05) and CAT (Figure 5(c), *p* < 0.01) were observed in the ISO group. XJEK (10 g/kg/d) and metoprolol treatment decreased MDA levels and increased endogenous antioxidants to normal levels.

### 3.5. XJEK Reduced the mRNA Expression of Atrial Natriuretic Peptide (ANP), Brain Natriuretic Peptide (BNP), *β*-Myosin Heavy Chain (*β*-MHC), and cTnI

ANP, BNP, and *β*-MHC are considered marker genes of myocardial hypertrophy. Compared with the control group, the expression of the ANP, BNP, and *β*-MHC mRNAs increased in the hearts of mice with MH and obviously decreased after XJEK (10 g/kg/d) and metoprolol treatment (Figures 6(a)–6(c), *p* < 0.05, *p* < 0.01). cTnI is an important indicator of the function of myocardial cells. Mice with MH presented increased cTnI expression; however, XJEK (10 g/kg/d) and metoprolol treatment markedly decreased the expression of the biochemical markers of myocardial damage (Figure 6(d), *p* < 0.05).

### 3.6. XJEK Alleviated Oxidative Stress in Mice with ISO-Induced MH by Modulating the Nrf-2/HO-1 Pathway

The nuclear expression of Nrf2 and its Nrf2-mediated antioxidant enzyme HO-1 was examined to explore the molecular mechanism underlying the protective effect of XJEK on OS in the heart. We noted increased total Nrf2, nuclear Nrf2, and HO-1 levels in mice with MH, but the differences were not statistically significant, while mice treated with XJEK and metoprolol exhibited significantly higher total Nrf2 and nuclear Nrf2 levels and markedly higher levels of HO-1, reflecting inactivation of the Nrf2 pathway (Figures 7(a)–7(e), *p* < 0.05). Similarly, an increase in the Nrf2 and HO-1 mRNA levels was observed following MH, and XJEK and metoprolol treatment resulted in significantly higher levels of the Nrf2 and HO-1 mRNAs (Figures 7(f)-7(g), *p* < 0.05, *p* < 0.01).

## 4. Discussion

Traditional Chinese medicine (TCM) has a history of thousands of years, has made an indelible contribution to the lives and reproduction of Chinese people, and has attracted worldwide interest [21]. XJEK is an effective clinical prescription with optimal efficacy. We previously used UPLC-Q-Extractive Orbitrap mass spectrometry to identify the main ingredients in XJEK, including *Panax ginseng* C. A. Mey, *Astragalus mongholicus* Bunge, *Polygonatum odoratum* (Mill.) Druce, and *Ophiopogon japonicus* (Thunb.) Ker-Gawl [22]. Studies have reported that these ingredients exert good therapeutic effects on cardiovascular diseases [23–25]. Additionally, we documented the ability of XJEK to inhibit cardiovascular remodeling in mice with high salt or L-name-induced hypertension [26–28]. Similarly, the present study showed that XJEK treatment significantly reduced myocardial hypertrophy and improved cardiac function in mice with ISO-induced MH, and a similar effect was observed for the positive drug metoprolol.

Though important advances in diagnosis and treatment for heart failure, its mortality rate has not significantly improved, and it is still one of the deadliest diseases worldwide. While the mechanisms for the occurrence and development of heart failure are not well understood, cardiac hypertrophy is believed one of them [29, 30]. Cardiac hypertrophy is featured by increased cell size, interstitial fibrosis, cell death, and cardiac dysfunction [31, 32]. This study demonstrated that HW/BW and LW/BW ratios, myocardial fibrosis, and the expressions of hypertrophic genes, ANP, BNP, and *β*-MHC, as well as the biomarker of myocardial injury, cTnI, were significantly increased by ISO treatment; while, XJEK and metoprolol reversed these changes. Data analyses from ECG and echocardiogram also showed that XJEK and metoprolol improved heart function in mice with ISO-induced MH. The pathogenesis of MH remains unclear, but the oxidative stress pathway is recognized as one of the classical underlying mechanisms of MH. Oxidative stress originating from an ISO injection is mediated primarily by *β*_1_-adrenergic receptors [33]. Stimulation of *β*_1_-adrenergic receptors rapidly generates ROS and decreases the total cellular antioxidant capacity. Adrenoceptor activation induced by ISO may be regulated by an oxidation mechanism. Significant changes in SOD, MDA, and GSH levels were observed in mice with ISO-induced MH [34]. In this study, mice with ISO-induced MH exhibited remarkably increased levels of MDA and decreased SOD and CAT levels, consistent with previous studies. The Nrf2/HO-1 pathway is the central regulator of cellular antioxidant responses [10]. Nrf2 is an intranuclear antioxidant that interacts with the downstream HO-1 protein after entering the nucleus to activate the oxidative stress pathway. As shown in the present study, the levels of proteins in the Nrf2/HO-1 pathway were slightly increased in the model group, presumably due to a self-protective mechanism, which may not be sufficient to resist heart injury. Treatment with XJEK at a high dose and metoprolol increased the expression of the protective oxidative products SOD and CAT while reducing MDA levels. Furthermore, RT-PCR and Western blot analyses indicated that the nuclear translocation of Nrf2 and the expression levels of HO-1 were increased significantly following high-dose XJEK and metoprolol administration. Therefore, the present study suggested that the antioxidant activity of XJEK may activate the Nrf2/HO-1 pathway via the upregulation of Nrf2.

## 5. Conclusions

In summary, marked OS, cardiac remodeling, and cardiac dysfunction were observed in ISO-treated mice and were reversed by XJEK and metoprolol treatments. The protective effects of XJEK on mice with ISO-induced MH may be related to the activation of the Nrf2/HO-1 signaling pathway. Further detailed studies are required to fully clarify the underlying mechanisms.

## Figures and Tables

**Figure 1:** Effects of XJEK on HW/BW and LW/BW in mice with ISO-induced MH. (a) Representative figure of heart macroscopic images. (1) Control group; (2) model group; (3) 7.5 g/kg XJEK+ISO-treated group; (4) 10 g/kg XJEK+ISO-treated group; (5) metoprolol+ISO-treated group. (b) HW/BW, heart to body weight. (c) LW/BW, lung to body weight. Data are presented as the means ± SD, *n*  =  8. ^*∗*^*P* < 0.05 and ^*∗∗*^*P* < 0.01 compared with the control group; ^#^*P* < 0.05 and ^##^*P* < 0.01 compared with the model group.

**Figure 2:** Effects of XJEK on myocyte CSA and fibrotic area in mice with ISO-induced MH. (a)-(b) Representative images of myocyte CSA and the long axis (HE staining; magnification×200). (c) Representative images of myocardial fibrosis (Masson's trichrome staining;). Statistical analysis of the (d) myocyte CSA (cross-sectional area) and (e) fibrotic area in the injured heart. (1) Control group; (2) model group; (3) 7.5 g/kg XJEK + ISO-treated group; (4) 10 g/kg XJEK+ISO-treated group; (5) metoprolol+O-treated group. Data are presented as the means ± SD, *n* = 8. ^*∗∗*^*P* < 0.01 compared with the control group; ^##^*P* < 0.01 compared with the model group.

**Figure 3:** ECG recordings and depiction of the ECG parameters measured. (a) Representative images of ECG in different groups of mice. (A-1) Control group; (A-2) model group; (A-3) 7.5 g/kg XJEK + ISO-treated group; (A-4) 10 g/kg XJEK + ISO-treated group; (A-5) metoprolol+ISO-treated group. Statistical analysis of the (b) heart rate, (c) R amplitude, and (d) QT interval. Data are presented as the means ± SD, *n* = 8. ^*∗∗*^*P* < 0.01 compared with the control group; ^#^*P* < 0.05 and ^##^*P* < 0.01 compared with the model group.

**Figure 4:** Echocardiogram recordings and derived echocardiographic parameters in mice. (a): Representative images of echocardiogram in different groups of mice. (A-1): Control group; (A-2): model group; (A-3): 7.5 g/kg XJEK + ISO-treated group; (A-4): 10 g/kg XJEK + ISO-treated group; (A-5): metoprolol+ISO-treated group. (b) EF, ejection fraction. (c) FS, fractional shortening of the left ventricular diameter. (d) LVESv, left ventricular volume at end-systole. (e) LVIDs, left ventricular diameter at end-systole. (f) LVPWd, left ventricular posterior wall thickness at end-diastole. (g) LVPWs and left ventricular posterior wall thickness at end-systole. Data are presented as the means ± SD, *n* = 8. ^*∗*^*P* < 0.05 and ^*∗∗*^*P* < 0.01compared with the control group; ^#^*P* < 0.05, ^##^*P* < 0.01 compared with the model group.

**Figure 5:** Effects of XJEK on serum MDA (a), SOD (b), and CAT (c) levels in mice with ISO-induced MH. Data are presented as the means ± SD, *n* = 8. ^*∗*^*P* < 0.05 and ^*∗∗*^*P* < 0.01 compared with the control group; ^#^*P* < 0.05 and ^##^*P* < 0.01 compared with the model group.

**Figure 6:** XJEK treatment reduced the mRNA expression levels of ANP (a), BNP (b), *β*-MHC (c), and cTnI (d) in heart tissues. Data are presented as the means ± SD, *n* = 3. ^*∗*^*P* < 0.05 and ^*∗∗*^*P* < 0.01 compared with the control group; ^#^*P* < 0.05 and ^##^*P* < 0.01 compared with the model group.

**Figure 7:** Effects of XJEK treatment on the nuclear translocation of Nrf2 and HO-1 expression in heart tissues from mice with MH. The expression levels of Nrf2 and HO-1 in heart tissues examined using Western blot analysis (a)–(e) and RT-PCR (f)-(g). Data are presented as the means ± SD, *n* = 3. ^*∗*^*P* < 0.05 compared with the control group; ^#^*P* < 0.05 and ^##^*P* < 0.01 compared with the model group.

**Table 1:** Recipe of XJEK formulation.

Components	Voucher specimens number	Part for use	Rate (%)
*Panax ginseng* C. A. Mey	PCAHMU-20121005	Root	11.71
*Polygonatum odoratum* (Mill) Druce	PCAHMU-20121006	Rhizome	7.03
*Panax pseudoginseng* var. *notoginseng* (Burkill) G. Hoo and C. L. Tseng	PCAHMU-20121007	Root	3.09
*Allium macrostemon* Bunge	PCAHMU-20121008	Ramulus	7.80
*Angelica sinensis* (Oliv.) Diels	PCAHMU-20121009	Root	7.80
*Ophiopogon japonicus* (Thunb.) Ker-Gawl.	PCAHMU-20121010	Root	7.80
*Schisandra chinensis* (Turcz.) Baill.	PCAHMU-20121011	Fruit	3.93
*Salvia miltiorrhiza* f. alba C. Y. Wu and H. W. Li	PCAHMU-20121012	Root	7.80
*Sophora flavescens* Aiton	PCAHMU-20121013	Root	7.80
*Glycyrrhiza acanthocarpa* (Lindl.) J. M. Black	PCAHMU-20121014	Rhizome	7.80
*Astragalus* mongholicus Bunge	PCAHMU-20121015	Root	11.69
Epimedium *acuminatum* Franch	PCAHMU-20121016	Aerial part	7.80
*Trichosanthes obtusiloba* C. Y. Wu	PCAHMU-20121017	Seed	7.80
*Dryobalanops aromatica* C. F. Gaertn	PCAHMU-20121018	Resin	0.15

**Table 2:** Primer sequences used for real-time quantitative RT-PCR.

Target gene	Forward primer (5′-3′)	Reverse primer (5′-3′)	Product length (bp)
ANP	GGTCTAGTGGGGTCTTGCCTCTC	GCGTCTGTCCTTGGTGCTGAAG	114
BNP	TGGGCTGTAACGCACTGAAGTTG	AGAGACCCAGGCAGAGTCAGAAAC	81
*β*-MHC	CACCAGCCTCATCAACCAGAAGAAG	TCCTCTGCGTTCCTACACTCCTG	99
cTnI	AGGAGATGGAACGAGAGGCAGAAG	CGTGAAGCTGTCGGCATAAGTCC	129
Nrf2	AAGCACAGCCAGCACATTCTCC	TGACCAGGACTCACGGGAACTTC	130
HO-1	ACCGCCTTCCTGCTCAACATTG	CTCTGACGAAGTGACGCCATCTG	104
GAPDH	GGTTGTCTCCTGCGACTTCA	TGGTCCAGGGTTTCTTACTCC	183

## Data Availability

The data used to support the findings of this study are available from the corresponding author upon request.
